# CT Image Features under Reconstruction Algorithm in Analysis of the Effect of Probiotics Combined with Ursodeoxycholic Acid in Treatment of Intrahepatic Cholestasis of Pregnancy

**DOI:** 10.1155/2021/1709793

**Published:** 2021-10-31

**Authors:** Hongxue Liu, Haidong Wang, Muling Zhang

**Affiliations:** Department of Obstetrics, The Affiliated Huaian No. 1 People's Hospital of Nanjing Medical University, Huai'an 223300, Jiangsu, China

## Abstract

This research was to explore the adoption value of computed tomography (CT) images based on adaptive statistical iterative reconstruction (ASIR) algorithm in the evaluation of probiotics combined with ursodeoxycholic acid in the treatment of intrahepatic cholestasis of pregnancy (ICP). A total of 82 patients with ICP were selected as the research subjects and they were randomly rolled into experimental group (380 mg probiotics enteric-soluble capsule twice a day, combined with 90 mg ursodeoxycholic acid soft capsule three times a day) and control group (90 mg ursodeoxycholic acid soft capsule three times a day), with 41 cases in each. The treatment course was four months. The ASIR algorithm was constructed and applied to the CT image analysis and diagnosis of ICP patients. The effects of filtering back projection (FBP) reconstruction and ASIR algorithm on CT image quality, denoising degree, and artifacts of ICP patients were compared. Moreover, blood indicator levels of ICP patients before and after treatment were assessed. The results showed that the SD values of liver and gallbladder (20.77 Hu and 27.58 Hu) in the reconstructed image of the ASIR algorithm were significantly lower than those of the FBP algorithm (40.58 Hu and 45.63 Hu) (*P* < 0.05). The SNR values of the liver and gallbladder (3.68 and 2.05) of the reconstructed image were significantly higher than those of the FBP algorithm (1.91 and 1.19) (*P* < 0.05). The overall image quality after ASIR reconstruction (3.92 points) was significantly better than that of the FBP algorithm (2.36 points), and the image noise score (3.21 points) reconstructed by the FBP algorithm was higher than that by the ASIR algorithm (1.83 points). The artifact score of FBP reconstructed image (4.47 points) was greatly higher than that of ASIR algorithm (2.26 points) (*P* < 0.05). Before treatment, there was no remarkable difference in the indexes between the two groups of patients (*P* > 0.05). After treatment, the *γ*-glutamyltransferase (*γ*-GT) and alkaline phosphatase (ALP) levels (327.55 U/L and 778.15 *μ*mol/L) of the experimental group of ICP patients were higher than those of the control group (248.63 U/L and 668.43 *μ*mol/L), with substantial difference between the two groups (*P* < 0.05). The blood ammonia (BA) level (151.09 *μ*mol/L) of the experimental group was lower than that of the control group (178.46 *μ*mol/L), and the difference between the two groups was remarkable (*P* < 0.05). To sum up, the CT image denoising degree based on ASIR algorithm was high, with few artifacts and good overall quality. Probiotics combined with ursodeoxycholic acid in the treatment of ICP can effectively improve the liver function and intestinal flora of patients, which was of great significance in the clinical diagnosis and treatment of the disease.

## 1. Introduction

Intrahepatic cholestasis of pregnancy (ICP) is a female disease occurring during pregnancy, which will endanger the fetus and lead to the increase of neonatal morbidity and mortality [1]. Patients with ICP typically experience problems such as elevated blood and bile acids and abnormal liver function. For pregnant women, these symptoms usually disappear immediately after delivery, but they are harmful to the fetus, and fetal intrauterine compression causes premature delivery, leading to neonatal asphyxia or death [2]. The incidence of this disease is up to 0.8%–12.0%, and it disappears immediately after delivery. However, the recurrence rate is high, and the patients will relapse again when they become pregnant again or take contraceptive drugs [3]. The pathogenesis of ICP is complex and not yet clear. Treatment is mainly through choleretics and hepatoprotective drugs, such as ursodeoxycholic acid and choline [4]. At present, researchers usually combine adenosylmethionine with ursodeoxycholic acid for research, but there are some shortcomings such as small sample size and complex control. Studies pointed out that probiotics can improve the microecological environment in vivo, with low cost and no invasion, which can prevent and cure hepatobiliary diseases and reduce the harm [5]. At present, there are few studies combining ursodeoxycholic acid and probiotics to treat IPC.

Nowadays, computed tomography (CT) is widely utilized in clinical medicine. Because of its fast scanning speed and clear images, it has become the main imaging tool for medical auxiliary diagnosis and scientific research. CT liver scan can choose any time phase for continuous scan. After a lot of clinical practice, CT scan has become a routine method for examination of liver and gallbladder diseases, and it has played an important role in the diagnosis and treatment of IPC [6]. The CT image reconstruction method is an important technology in the image imaging process, and the optimization of the image is particularly important. At present, the filtered back projection (FBP) method is the main algorithm for CT image reconstruction. The algorithm reconstructs quickly, but the noise is obvious, the imaging is not detailed enough, and it will aggravate the patient's radiation. The iterative reconstruction (IR) algorithm also has problems such as noise and artifacts [7]. Adaptive statistical iterative reconstruction (ASIR) can improve imaging quality, reduce radiation dose, and overcome the shortcomings of the above technologies, which is the most widely utilized iterative reconstruction technology at present [8]. ASIR image reconstruction algorithm can reduce imaging noise and artifact, improve image quality without interfering with clinical diagnosis, and is utilized for clinical treatment, which has been approved by the American medical management system [9]. In this study, ICP patients were taken as the research object, and the ASIR algorithm was applied to the CT image analysis and diagnosis of ICP patients by constructing the ASIR algorithm. The effects of filtering back projection (FBP) reconstruction and ASIR algorithm on CT image quality, denoising degree, and artifacts of ICP patients were compared. Blood indicator levels of ICP patients before and after treatment were detected to evaluate the clinical effect of probiotics combined with ursodeoxycholic acid in ICP treatment. It was hoped to provide a reliable basis for the application of ASIR based CT imaging in clinical diagnosis and treatment.

## 2. Materials and Methods

### 2.1. Research Objects

A total of 82 patients, ranging in age from 24 to 36 years, with an average age of 26 years, who underwent ICP specific detection in our hospital from July 2019 to May 2020, were selected for CT imaging examination. They were randomly divided into experimental group and control group, with 41 patients in each group. There was no statistical difference in general information between the two groups (*P* > 0.05). This study had been approved by the Ethics Committee of the Hospital, and informed consent was signed by the patients and their families.

Inclusion criteria were as follows: (i) clinically confirmed ICP patients (the ICP diagnostic criteria of *Chinese Journal of Obstetrics and Gynecology* edited by Cao [10]); (ii) skin pruritus being the main symptom during pregnancy; (iii) abnormal liver function, mainly slightly increased serum transaminase; (iv) the patient being in good general condition without obvious vomiting, weakness, or other diseases; (v) pruritus quickly subsiding after delivery, and liver function quickly returning to normal; and (vi) patients with elevated bile acid level.

Exclusion criteria for subjects were as follows: (i) those who had liver or gallbladder disease, or skin diseases before pregnancy which affected the observation indicators; (ii) patients who had received treatment that affected the observation indicators before inclusion; (iii) only statistical results without specific data listed; (iv) those who utilized the combination of drugs which affected the judgment of the results and could not be excluded by the control.

### 2.2. Grouping

The included IPC patients were randomly divided into experimental group and control group, with 41 patients in each group. Patients in the experimental group were given probiotic enteric-coated capsules 380 mg twice a day, combined with ursodeoxycholic acid soft capsules 90 mg three times a day for four months. Patients in the control group were given ursodeoxycholic acid soft capsule 90 mg three times a day for four months. During the treatment, neither group of patients took other drugs.

### 2.3. Observation Indicators and Detection

The blood sample test was as follows: 5 mL of venous blood was extracted from the patients on an empty stomach in the morning and placed in an anticoagulant tube. Levels of *γ*-glutamyl transferase (*γ*-GT), blood ammonia (BA), alkaline phosphatase (ALP), and total cholesterol (TC) were detected by Hitachi automatic biochemical analyzer.

### 2.4. Inspection Method and Reconstruction Method

All patients were scanned using a General Electric 256-bar wide-body detector CT (Revolution, General Engine, GE, USA). Prior to the CT scan, the patients underwent inhalation and breath-holding training to reduce breathing movements and removed clothing at the site of examination, including various items with metallic substances, such as earrings and keys. During the examination, the patients were supine with their arms raised above their heads, and they were required not to move freely to avoid artifacts. Patients were first examined with a conventional dose scan, with a preset noise index (NI) of 14. FBP was utilized for image reconstruction. The NI was set at 24, and the image was reconstructed by ASIR. Scanning was under 120 KV and 150 mAs, reconstruction layer thickness was 0.625 mm, field of view was 220 mm, scanning time was 0.5 s, cycle time was 1 s, and matrix was 512 × 512.

### 2.5. CT Image Reconstruction Based on ASIR Algorithm

The main idea of the ASIR iterative reconstruction algorithm is making all currently estimated images satisfy an equation in each update. In the iterative correction process, only the projection value of one projection unit is considered at a time. The calculation process of the reconstruction algorithm is shown in Figure 1.

The specific reconstruction steps of the ASIR algorithm are as follows:

(I) Assign an unknown image vector, and *k* is a constant.
  (1) $$\begin{array}{c} R_{k}=R_{k}{}^{\left(0\right)}\left(k=1,2,3...n\right). \end{array}$$
(II) The estimated projection values of all equations are calculated, where *Z*_*kc*_ is the relaxation parameter.
  (2) $$\begin{array}{c} Y_{c}{}^{*}=\sum_{k=1}^{n}Z_{kc}R_{k}{}^{\left(0\right)}\left(k=1,2,3...n\right). \end{array}$$
(III) The error is calculated, and **Φ** is the error parameter.
  (3) $$\begin{array}{c} \Phi_{c}=Y_{c}-Y_{c}{}^{*}\left(k=1,2,3,...n\right). \end{array}$$
(IV) The correction value of the *k*-th pixel is calculated.
  (4) $$\begin{array}{c} E_{k}=\frac{1}{Z_{kc}}\sum_{k=1}^{N}\Phi_{c}\frac{1}{Z_{ik}}. \end{array}$$
Among them, *i* is the ray passing through pixel *k*, and all rays passing through the pixel are summed at the same time.
(V) The *k*-th pixel value is corrected.
  (5) $$\begin{array}{c} R_{k}=E_{k}+R_{k}{}^{\left(0\right)}. \end{array}$$
To sum up, all rays passing through the pixel are utilized to correct it to complete the first iteration. The average value of each projection band can reduce the error, thereby avoiding the influence caused by the reconstruction result, which has a noise reduction effect in the image reconstruction process.

### 2.6. Image Objective and Subjective Evaluation Indicators

After reconstruction, two kinds of noise reduction images of each patient were obtained, and all the images were transmitted to GE workstation (General Engine Advantage Workstation 4.7). The patient's personal information and scan and reconstruction information were hidden. The patient's CT value (the relative density of tissue structure on the CT image, in Hu) and the SD value (the background noise value of the abdominal fat on the same plane) were measured. The signal-to-noise ratio (SNR) was calculated. SNR = CT value/SD value. All data were measured three times, and the average value was taken as the final statistical result.

Subjective evaluation was performed by radiologists using a double-blind method to evaluate all images. A 5-point system was adopted to evaluate the overall image quality (unclear texture, blurred contrast, and unclear image indicated 1 point; the texture was fuzzy, the contrast was fuzzy, and the image roughly indicated 2 points; the texture was not clear, the contrast was not clear, and the image was not fine, indicating 3 points; the texture was clear, the contrast was clear, and the image was delicate, indicating 4 points; clear texture, clear contrast, and fine image indicated 5 points). A 5-point Likert method [11] was adopted to evaluate image noise (image noise was completely acceptable, 1 point; less than average noise, 2 points; average noise, 3 points; above average noise, 4 points; unacceptable image noise, 5 points). Each artifact was also scored by a 5-point method (no artifact, 1 point; small artifacts did not affect the organizational structure, 2 points; slight effects on the structure, 3 points; the artifact was large, affecting the main structure, 4 points; the artifact was extremely heavy, and the image was unacceptable, 5 points).

### 2.7. Statistical Analysis

SPSS 24.0 was utilized for statistical analysis. All experimental data were represented as mean ± standard deviation ($\bar{x}$ ± s). One-way analysis of variance was utilized for statistical data. Friedman rank-sum test was utilized to compare the subjective scores of overall image quality, noise, and artifacts, and the test level was *α* = 0.05. *P* < 0.05 was statistically remarkable.

## 3. Results

### 3.1. Abdominal CT Images of ICP Patients with Different Reconstruction Algorithms

Figure 2 shows a 28-year-old ICP patient with a thin-slice CT scan of the lower abdomen with two reconstruction algorithms. A, B, and C represent the plain scan phase, arterial phase, and portal phase, respectively, and A1, B1, and C1 represent FBP, while A2, B2, and C2 represent ASIR. Observed from the CT image, the image reconstructed by the ASIR algorithm shows that the lesion area is relatively clear, and the edge contrast is high. The FBP reconstructed image has blurry edges and poor contrast. The overall quality of the FBP reconstructed image is worse than that of ASIR, the image noise is high, and the artifacts are obvious.

### 3.2. Objective Indicator Analysis of CT Image Based on Reconstruction Algorithm

Routine CT scans of the abdomen of 30 ICP patients were performed, and the initial images were reconstructed by two reconstruction algorithms, FBP and ASIR. The unreconstituted images with a thickness of 0.625 mm were obtained. According to the obtained images, the data of different organs in the abdomen of ICP patients were measured and analyzed, and the CT, SD, and SNR values of the reconstructed image under different reconstruction algorithms were obtained.

#### 3.2.1. CT Value Analysis of Reconstructed Image

The CT value analysis results are shown in Figure 3. For the CT value of the liver, the CT values of the reconstructed image of FBP and ASIR were 77.43 Hu and 76.51 Hu, respectively, and there was no considerable difference between the two (*P* > 0.05). For the CT value of the gallbladder, the CT values of the reconstructed images of FBP and ASIR were 54.37 Hu and 56.58 Hu, respectively, and the difference between the two was not remarkable (*P* > 0.05).

#### 3.2.2. SD Value Analysis of Reconstructed Image

The SD value analysis results are shown in Figure 4. The SD value of the liver was analyzed. The SD values of the reconstructed image of the FBP and ASIR algorithms were 40.58 Hu and 20.77 Hu, respectively. The SD value of the reconstructed image of the ASIR algorithm was notably lower than that of the FBP algorithm (*P* < 0.05). The SD value of the gallbladder was analyzed. The SD values of the reconstructed image of FBP and ASIR were 45.63 Hu and 27.58 Hu, respectively. The SD value of the reconstructed image of the ASIR algorithm was notably lower than that of the FBP algorithm (*P* < 0.05).

#### 3.2.3. SNR Value Analysis of Reconstructed Image

The SNR value analysis results are shown in Figure 5. The SNR value of the liver was analyzed. The SNR values of the reconstructed image of the FBP and ASIR algorithms were 1.91 and 3.68, respectively. The SNR value of the reconstructed image of the ASIR algorithm was notably lower than that of the FBP algorithm (*P* < 0.05). The SNR value of the gallbladder was analyzed. The SNR values of the reconstructed image of the FBP and ASIR algorithms were 1.19 and 2.05, respectively. The SNR value of the reconstructed image of the ASIR algorithm was notably lower than that of the FBP algorithm (*P* < 0.05).

In summary, in the CT image of the ASIR algorithm, the noise value (SD value) of the abdominal liver and gallbladder of ICP patients was notably lower than that of the FBP reconstruction algorithm, while the signal-to-noise ratio (SNR) was considerably higher than that of the FBP reconstruction image. There was no considerable difference in the CT value of the reconstructed image between the two algorithms.

### 3.3. Subjective Evaluation of CT Images Based on Reconstruction Algorithm

Figures 6 and 7 show partially enlarged views of CT images of a certain ICP patient's abdominal CT reconstructed by FBP and ASIR, respectively.

Figure 8 shows the mean statistical graph of the overall quality, noise, and artifacts of the reconstructed CT image scored by the radiologist. The scoring results showed that the image quality scores of the FBP and ASIR algorithms were 2.36 and 3.92, respectively. The overall image quality after ASIR reconstruction was substantially better than that of the FBP algorithm (*P* < 0.05). In the evaluation of image noise, the scores of FBP and ASIR were 3.21 and 1.83, respectively. Compared with the ASIR algorithm, the FBP reconstructed image had higher noise, and the difference was remarkable (*P* < 0.05). The evaluation of image artifacts showed that FBP had more image artifacts than the ASIR algorithm, and the difference was remarkable (*P* < 0.05).

### 3.4. Observation Indicators of Experimental Group and Control Group before and after Treatment

The ICP patients in the experimental group were treated with probiotics combined with ursodeoxycholic acid, and the ICP patients in the control group were treated with ursodeoxycholic acid. The blood indicators of the two groups of patients before and after treatment were recorded, including *γ*-glutamyl transferase (*γ*-GT), blood ammonia (BA), alkaline phosphatase (ALP) levels, and total cholesterol (TC). The changes of these indicators were analyzed to draw a graph of the changes of blood indicators in each group before and after treatment. The results showed that, before treatment, there was no statistical difference in each indicator between the two groups of patients (*P* > 0.05). After treatment, the *γ*-GT and ALP levels of ICP patients in the experimental group were higher than those in the control group, and the difference was remarkable (*P* < 0.05). The BA level of the experimental group greatly was lower than that of the control group (*P* < 0.05). The difference in TC values between the two groups after treatment was not remarkable (*P* > 0.05).  Figure 9 shows a graph of the changes of blood indicator levels before and after treatment in the experimental group and the control group.

## 4. Discussion

ICP generally has familial clusters, and the rate of recurrence is high. Medically, it is generally treated with liver protection and choleretic treatment [1]. The liver and gallbladder in the human body and the gastrointestinal system have the same embryonic origin, so there is a close relationship between tissue composition and organic function [12]. Probiotics can improve the microecological environment in the body, are cheap and noninvasive, which can prevent and treat liver and gallbladder diseases, reduce harm, and are nonpathogenic. Ursodeoxycholic acid can induce the massive secretion of endogenous bile acid in the treatment of IPC, regulate the concentration of hydrophilic bile acid, and prevent the functional damage of liver cells in the body. In this way, the liver's blocking structure is adjusted to alleviate the degree and progression of IPC patients [13].

This study combined probiotics and ursodeoxycholic acid to treat IPC. The results showed that, before treatment, there was no statistical difference in each indicator between the two groups of patients (*P* > 0.05). After treatment, the *γ*-GT and ALP levels of ICP patients in the experimental group were greatly higher than those in the control group (*P* < 0.05). The BA level of the experimental group was lower than that of the control group, and the difference was remarkable (*P* < 0.05). There was no considerable difference in TC values between the two groups after treatment (*P* > 0.05). It was proved that the combined application of ursodeoxycholic acid and probiotics was effective in improving liver function in patients with ICP, which may be related to the antioxidant and antiapoptotic effects of ursodeoxycholic acid in the above-mentioned mechanism [14]. Probiotics can regulate the intestinal flora, avoid excessive growth of small intestinal bacteria, and reduce intestinal endotoxemia and BA levels. They can also improve the liver function of patients and reduce the occurrence of mild HE and the possibility of mild HE progressing to clinical symptoms of HE [15]. There were no adverse reactions in all cases in this study, which also suggested that the drug had good safety.

Nowadays, CT is widely utilized in clinical medicine. Because of its advantages such as fast scanning speed and clear images, it has become the main imaging tool for medical auxiliary diagnosis and scientific research, which has played an important role in the diagnosis and treatment of IPC [16]. FBP, which is often utilized in image inspection, has heavy artifacts, great noise, and insufficient image quality [17]. ASIR can improve the image quality, reduce the radiation dose, and overcome the shortcomings of the above technologies and is currently the most widely utilized iterative reconstruction [18]. ASIR uses the resources obtained by FBR as the initial image for reconstruction, changes the measured values of different pixels into new estimated values, and then compares the target value with the new value. In the subsequent iterative reconstruction, the process is repeated until the new pixel value is wirelessly close to the expected value [19]. In recent years, iterative reconstruction has gradually been introduced into the field of image noise reduction. A series of current studies have also observed that ASIR has better image quality than FBP [20]. In this study, the subjective evaluation results of CT images showed that, in terms of image quality, the scores of FBP and ASIR were 2.36 and 3.92, respectively. The overall image quality after ASIR reconstruction was substantially better than that of the FBP algorithm (*P* < 0.05). In the evaluation of image noise, the scores of FBP and ASIR were 3.21 and 1.83, respectively. Compared with the ASIR algorithm, the FBP reconstructed image had higher noise, and the difference between the two was remarkable (*P* < 0.05). In the evaluation of image artifacts, FBP had more image artifacts than ASIR algorithm reconstruction, and the difference was remarkable (*P* < 0.05). It was shown that the image noise of ASIR at the aorta and skeletal muscle was notably lower than that of traditional FBP and ASIR, and the image quality can meet clinical needs. The objective indicator analysis results of the CT image showed that, in the CT image of the ASIR algorithm, the noise value (SD value) of the abdominal liver and gallbladder of ICP patients was notably lower than that of the FBP reconstruction algorithm (*P* < 0.05). However, the SNR was considerably higher than the FBP reconstructed image (*P* < 0.05). These results were consistent with the research conclusions of Dimmitt et al. (2019) [21]. It was proved that the noise of the CT image reconstructed by the ASIR model was considerably reduced, the image quality was improved, and the advantages of image quality and lesion detection were obvious.

## 5. Conclusion

In this study, patients with intrahepatic cholestasis of pregnancy (ICP) were selected as the research objects. ASIR reconstruction algorithm was established, which was applied to the CT image analysis and diagnosis of ICP patients, and the influence of the reconstruction algorithm on the CT image of ICP patients was discussed. Then, the clinical effect of probiotics combined with ursodeoxycholic acid in the treatment of ICP was evaluated. The results showed that SD and SNR values of liver and gallbladder reconstructed by ASIR algorithm were significantly lower than those of FBP algorithm. The overall image quality, image noise score, and pseudofilm review score after ASIR reconstruction were significantly better than those of FBP algorithm (*P* < 0.05). Before treatment, there was no statistical difference in all indicators between the two groups (*P* > 0.05). After treatment, the levels of *γ* -glutamyl transferase (*γ*-GT) and alkaline phosphatase (ALP) in the experimental group were higher than those in the control group, while the level of serum ammonia (BA) in the experimental group was lower than that in the control group, both with substantial differences (*P* < 0.05). It was proved that CT images based on ASIR reconstruction algorithm had high denoising degree, fewer artifacts, and good overall quality. Probiotics combined with ursodeoxycholic acid in the treatment of ICP can effectively improve the liver function and intestinal flora of patients. This study can provide a reliable basis for the adoption of CT imaging technology based on ASIR reconstruction algorithm in the diagnosis and treatment of ICP. However, the deficiency is that only abdominal CT images based on ASRI reconstruction algorithm at conventional doses are discussed. In future clinical studies, the influence of ASRI reconstruction algorithm on low-dose CT images needs to be discussed, so as to further illustrate its noise reduction efficiency in CT images.

## Figures and Tables

**Figure 1:** Schematic diagram of the calculation process of ASIR iterative reconstruction algorithm.

**Figure 2:** FBP and ASIR reconstruction of the CT scan of the abdomen of ICP patients. A, B, and C represent the plain scan phase, arterial phase, and portal phase, respectively, and A1, B1, and C1 represent FBP, while A2, B2, and C2 represent ASIR.

**Figure 3:** CT values of reconstructed images.

**Figure 4:** SD values of reconstructed images. ^*∗*^indicates that the SD value of the reconstructed image of FBP and ASIR algorithm is substantially different (*P* < 0.05).

**Figure 5:** SNR values of reconstructed images. ^*∗*^indicates that the SNR value of the reconstructed image of FBP and ASIR algorithm is substantially different (*P* < 0.05).

**Figure 6:** The partially enlarged views of liver imaging after reconstruction of the abdominal CT image of an ICP patient in two ways. *Note.* The average scores of subjective evaluations of FBP reconstructed images show image quality of 2.34 points, noise of 2.33 points, and artifacts of 4.45 points; the average scores of subjective evaluations of ASIR reconstructed images show image quality of 3.9 points, noise of 1.85 points, and artifacts of 2.34 points.

**Figure 7:** The partially enlarged views of gallbladder imaging after reconstruction of the abdominal CT image of an ICP patient in two ways. *Note.* The average scores of subjective evaluations of FBP reconstructed images show image quality of 2.38 points, noise of 2.29 points, and artifacts of 4.49 points; the average scores of subjective evaluations of ASIR reconstructed images show image quality of 3.94 points, noise of 1.81 points, and artifacts of 2.38 points.

**Figure 8:** Subjective scoring results of reconstructed images. *Note.*^*∗*^ indicates that the subjective scores of the reconstructed images of FBP and ASIR algorithms are substantially different (*P* < 0.05).

**Figure 9:** Changes of blood indicators in the experimental group and the control group before and after treatment. (a) The changes of *γ*-GT in the two groups of patients, (b) the changes in BA of the two groups of patients, (c) the changes in ALP of the two groups of patients, and (d) the changes in TC of the two groups of patients. ^*∗*^indicates considerable differences in blood indicators between the experimental group and the control group (*P* < 0.05).

## Data Availability

The data used to support the findings of this study are available from the corresponding author upon request.
